# Tamoxifen Prevents Peritendinous Adhesions: A Preliminary Report

**DOI:** 10.1155/2022/4250771

**Published:** 2022-09-20

**Authors:** Oguz Kayiran, Suphan Tunc, Guler Gamze Eren Ozcan, Neslihan Kaya, Derya Karabulut

**Affiliations:** ^1^Department of Plastic, Reconstructive and Aesthetic Surgery, Demiroglu Bilim University, Turkey; ^2^Private Practice in Plastic, Reconstructive and Aesthetic Surgery, Turkey; ^3^Department of Pathology, Sultan Abdulhamid Han Training and Research Hospital, Turkey; ^4^Department of Mechanical Engineering, Istanbul University, Turkey

## Abstract

**Background:**

Scarless healing comprises the ultimate goal after an injury. Since tendon healing results in a fibrotic scar, an injured tendon can never regain the mechanical potential and strength of its uninjured form. A wide variety of studies focus on the tendon healing with an absent or minimal peritendinous adhesions. However, no simple method has managed it at all. Possible complex actions and peritendinous environmental events take place during the tendon healing process. Tamoxifen (TAM), besides its breast cancer-related usage, is a potent antifibrotic drug. Here, we aimed to reduce the peritendinous adhesion with TAM administration.

**Methods:**

Achilles tendons of 44 Wistar albino rats were randomly distributed in 4 groups. In group 1, bilateral lower extremities were used as control and sham. Groups 2 and 3 were comprised of low-dose (1 mg/kg) and high-dose (40 mg/kg) systemic administration of TAM, respectively. Group 4 included local administration (1 mg/kg) of TAM. Biomechanical, macroscopical, and histopathological analyses were done and compared statistically. Biomechanically, the maximum force that led to tendon rupture was determined, and tensile force data were recorded via tensile testing device. Macroscopical and histopathological analysis were composed of the quantity, quality, and grade of peritendinous adhesions.

**Results:**

Macroscopic and histopathologic findings revealed that groups 2 and 3 had a variety of values ranging between slight to severe adhesions. In group 2, almost half of the animals had moderate adhesions, whereas in group 3, the majority of the animals had moderate adhesions. There were no animals with moderate or severe adhesions in group 4. Statistically significant values were calculated between sham and control groups. Biomechanically, group 2 showed the most significant result. The tendons in group 2 had the highest stiffness when maximal force was applied to rupture the tendons. Henceforth, all these consequences were proven statistically.

**Conclusion:**

We achieved less peritendinous adhesion with the local administration of TAM when compared to systemic administration of TAM. A better understanding of the peritendinous environmental process will reveal to develop new therapies in the prevention of peritendinous adhesions.

## 1. Introduction

Tendon healing is a complex process that takes place via intrinsic and/or extrinsic mechanisms and consisted of 3 separate stages: inflammatory, fibroblastic or reparative, and remodeling [1–3]. The coordination between healing and limiting establishes the best outcome. Extrinsic healing occurs when the fibroblasts and inflammatory cells move in from outside the tendon and invade the healing site. In contrast, intrinsic healing occurs through the migration of cells from the endotenon and epitenon and has interference with the extrinsic healing. Typically, the extrinsic mechanism is activated earlier than the intrinsic mechanism and is thought to be responsible for the adhesion formation, whereas the intrinsic system is thought to help with collagen realignment and cross-linking [1].

Peritendinous adhesions can be a consequence of metabolic, traumatic, surgical, pharmacologic, and/or rheumatologic diseases [4–7]. Restrictive adhesions can alter the effect of tendon gliding and may eventually prevent a healthy movement. The main goal is to establish a good relationship between the tendon and the surrounding synovial sheath [8].

Literature welcomes various agents and materials in the prevention of adhesions [4, 8–10]. TAM is a synthetic nonsteroidal, antiestrogenic agent mainly used in the treatment and prevention of breast cancer [11]. Moreover, it has been shown to inhibit keloid fibroblast proliferation, reduce transforming growth factor-*β* (TGF-*β*), and diminish collagen production [11–13]. These effects take place via alteration of transcriptional synthesis, cellular proliferation, and the modulation of polypeptide growth factor production [14]. There are in vitro and in vivo studies evaluating the effects of TAM. Recently, the beneficial effects of TAM on postoperative intra-abdominal adhesions were clarified [11]. However, the effects on peritendinous adhesions have never been elucidated.

In a recent study, the effects of TGF-*β* on tendon cell collagen production were clarified. Studies have shown the importance of TGF-*β* in flexor tendon healing [15–18]. Since TGF-*β* receptors are present in the tendon sheath, epitenon, and endotenon, modulation of TGF-*β* production could provide a mechanism to attenuate adhesion formation [15]. Therefore, here, the preventive effects of TAM on tendon gliding and postoperative adhesion are studied.

## 2. Material and Methods

Forty-four Wistar albino female rats, weighing 250 ± 25 g and 10-12 weeks of age, were included in the study [19]. They were housed in wire cages under constant temperature (21 ± 2°C) with a 12 h light-dark cycle and allowed free access to water and standard rat chow. This study was approved by the Local Animal Ethics Committee (2018-03/02) and performed under the National Guidelines for the Care and Use of Laboratory Animals.

All animals were anesthetized by intraperitoneal injection of 30 mg/kg ketamine hydrochloride (Ketalar, Parke-Davis, Istanbul) and 5 mg/kg xylazine (Rompun, Bayer, Istanbul). This experiment was conducted according to the animal model described by Zhang et al. [20] and Tosun et al. [21]. According to these models, Achilles tendons of the animals were used.

Under general anesthesia, in sterile conditions, a 2 cm incision was made above the proposed Achilles tendon. After the isolation of the tendon, the peritendon was transected with 15 scalpel. The suturation of the transected tendons was carried out with 4/0 polypropylene suture material using modified Kessler method.

The number of rats that will be used in the study was calculated according to power analysis via G-power. One-way ANOVA with 0.4 as effect size, 0.2 as alpha error, 0.8 as beta error, and 4 group study was conducted, and total sample size was found as 44. Forty-four rats were randomly divided into 4 groups:

Group 1 (*n* = 11): one lower extremity consisted of sham side (G1SHAM), and the other lower extremity of the same animal (contralateral) consisted of tendon isolation (Figure 1(a)), incision (Figure 1(b)), and repair (Figure 1(c)) with nonabsorbable suture material (control side=G1CON). Half of each lower extremity was used for biomechanical analyses, whereas the remaining half was sent to pathology

Group 2 (G2) (*n* = 11): tendon incision and repair with nonabsorbable suture material were carried out (Figure 1). Following the repair, 1 mg/kg TAM was administered daily via orogastric gavage for 4 weeks. One lower extremity of the animal was used for histopathological analyses and the other lower extremity of the same animal for biomechanical analyses

Group 3 (G3) (*n* = 11): the same as group 2 (Figure 1), but 40 mg/kg TAM was administered daily via orogastric gavage for 4 weeks. One lower extremity of the animal was used for histopathological analyses and the other lower extremity of the same animal for biomechanical analyses

Group 4 (G4) (*n* = 11): the same as group 2 (Figure 1), but 1 mg/kg TAM was locally injected daily to the repaired area for 4 weeks. One lower extremity of the animal was used for histopathological analyses and the other lower extremity of the same animal for biomechanical analyses

After the treatments, the skin incisions were closed with 4/0 polypropylene suture materials, and the legs were dressed and splinted. The animals were allowed unrestricted cage movements.

After 6 weeks, macroscopical, histopathological, and biomechanical analyses were conducted.

### 2.1. Histopathological Analysis

All samples were transferred to the pathology laboratory. By performing routine histopathological follow-up in the pathology laboratory, the samples were fixed with formalin and embedded in paraffin as blocks. Sections of 4-micron thickness were taken from these blocks and stained with hematoxylin and eosin (H&E). For Masson's trichrome staining, a section thickness of 3-5 microns is applied in the procedure. In our study, we wanted to take sections with the highest thickness so that the tissue would not be spilled, so we stained by taking 5 micron sections.

Paraffin blocks were cut 5 *μ*m sections and were stained with Masson's trichrome reagent to show collagen. Six drops of Weigert's iron hematoxylin-A solution and 6 drops of Weigert's iron hematoxylin-B solution were added to the slides and left for 10 minutes. Before the preparations were washed, 10 drops of picric acid alcoholic solution were dropped and left for 5 minutes and washed with distilled water. Afterwards, Ponceau acid fuchsin solution was dripped onto the slides and left for 15 minutes. Washing was done again with distilled water. Ten drops of phosphomolybdic acid solution were dripped onto the slides, left for 10 minutes, and washed. Finally, 10 drops of Masson's aniline blue were added and left for 10 minutes. It was washed in distilled water and quickly passed through alcohol. Then, the slides were covered with a coverslip after treatment with xylene.

All slides were evaluated with an Olympus BX-46 light microscope and photographed with an Olympus DP-72 camera by the same pathologist.

The macroscopic and microscopic adhesion criteria described by Tang et al. were used for macroscopic and histopathological evaluations in our study (Tables 1 and 2) [22]. Each tendon was given a score to feature the adhesions, macroscopically and histopathologically. Quantity (the length), quality (the density and the tolerance for mobility), and grade of adhesions were analyzed for each tendon and compared with the other groups to understand the effects of TAM. Mean macroscopic and histopathologic values were calculated to study the statistical test.

### 2.2. Biomechanical Test

Tendons were exposed to tension test for biomechanical examination. Tendons were delivered to Machine Materials Laboratory in Faculty of Mechanical Engineering in saline solution to prevent dehydration with a remarkable amount of bone from calcaneus on the distal side and muscle tissue on the proximal side.

The tensile testing device (Instron 5982, universal testing machine, Norwood, MA, USA; load capacity is 100 kN, speed range is 0.00005-50 mm/minute, sampling frequency is 1 kHz, and load measurement accuracy is ±0.5%) was used for all biomechanical tests. To mount the tendon specimens onto the tensile test machine, tendon-muscle and tendon-bone regions were securely fixed between sandpaper sheets which were then attached to the grips of the testing machine. Tendon-sandpaper contact was enabled by the adhesion of cyanoacrylate glues. Samples were stretched longitudinally with a constant speed of 6 mm/minute until they ruptured. Tensile force data were recorded, and the maximum force that led to tendon rupture was figured out (Figures 2(a) and 2(b)).

### 2.3. Statistical Analysis

Statistical analysis was calculated for each group of parameters such as macroscopic and histopathological findings and biomechanical findings. These analyses were performed using the IBM SPSS version 22.0 (IBM Corp., Armonk, NY, USA).

Dependent ordinal variables were checked for normality test. If not found as normal distributed, nonparametric tests were used to compare each dependent variable in one group with its related counterpart in another group.

Statistical analysis for macroscopic and histopathological findings: mean values were calculated for each group with the equivalent of the other group, and regarding the dependent ordinal variables, *p* below 0.05 was accepted as statistically significant according to the paired samples *t*-test

Statistical analysis for biomechanical findings: mean and standard deviation values were used to analyze descriptive data. Statistically significant difference with respect to each of the results obtained for each case was determined by ANOVA method. *p* below 0.01 was accepted as highly statistically significant.

## 3. Results

All animals survived at the end of the study. They were sacrificed at the end of the 6th week. No tendon ruptures or wound infection were noted.

### 3.1. Macroscopic and Histopathological (Microscopic) Findings

The tendons in group 1 control (G1CON) showed remarkable lengthening (quantity) and reduced tolerance and density to mobilize (quality) with significant consistence of peritendinous adhesions. Unsurprisingly, the tendons in group 1 sham (G1SHAM) did not show any of these findings. Macroscopically and microscopically, the mean quantity (macro1 and micro1 in the text and figures) and quality (macro2 and micro2 in the text and figures) parameters for all groups are calculated and shown in Table 3. According to these, groups 2 and 3 showed higher values than G1CON. On the contrary, group 4 manifested less values than G1CON.

Regarding adhesion scores, groups 2 and 3 had a variety of values ranging between slight and severe adhesions. In group 2, almost half of the animals had moderate adhesions, whereas in group 3, the majority of the animals had moderate adhesions. There were no animals with moderate or severe adhesions in group 4. Adhesion scores among the groups are calculated and shown in Table 3. Moreover, Table 4 summarizes the distribution of the number of the animals regarding their adhesion scores. Slight adhesion was established in group 4 which is similar with the control group. On the contrary, groups 2 and 3 had adhesions ranged between slight and severe.

Figure 3 summarizes histopathological findings among the groups.

According to the macroscopic and histopathological results, local administration of TAM (group 4) ensured similar pathological findings with the control group (G1CON).

### 3.2. Biomechanical Findings

Maximum force that led to tendon rupture was obtained in group 2 when compared to the other groups. This force was found to be minimum for the animals in group 3.  Figure 4 shows mean maximum rupture forces applied to the tendons and statistical significance among the groups.

The tendons in group 2 had the highest stiffness during maximal force. Following group 2, group 4 showed similar tensile strength with G1CON.

Biomechanical study showed that the tendons in group 2 had the highest values that led to rupture. Therefore, systemic administration of low-dose TAM ensured the best result among the other groups, biomechanically.

### 3.3. Statistical Findings

There was remarkable statistically significance difference between the control (G1CON) and sham (G1SHAM) groups, both for the macroscopic and microscopic parameters. Group 4 had the most significant values. Almost every parameter in group 4 revealed statistically significance when compared with the other groups. A detailed statistics can be seen on Table 5 and Figure 5.

Biomechanically, *p* value was calculated below 0.01 between G1CON and group 2 as well as G1SHAM and group 2. In addition, there were significant differences between G1SHAM and group 3, group 2 and group 3, group 2 and group 4, and group 3 and group 4, statistically.

Under these circumstances, group 4 had the upmost benefit in the reduction of peritendinous adhesions, pathologically. However, group 2 showed better biomechanical results. Thus, all these consequences were proven statistically.

## 4. Discussion

The ideal tendon repair has been described as one that has easy suture placement, secured knots, smooth end-to-end tendon alignment, minimal to no gapping at the repair site, avoiding injury to tendon vasculature, and allowing for early active mobilization [23–25]. The ultimate goal of surgical intervention has remained constant: to achieve enough strength to allow early motion, to prevent adhesions within the tendon sheath, and to restore the normal range of motion and function. Recently, research has focused on biological factors that will increase the tendon stability after surgical repair, enhance intratendinous healing, and decrease extratendinous fibrosis [20, 26, 27]. Additional research has clarified different suture configurations or number of core sutures to maximize the strength of tendon repair and postoperative rehabilitation protocols to maximize function [20, 28, 29]. Moreover, different suture materials and knot tying technique were used to approximate the tendons. Besides, FiberWire (Arthrex, Naples, FL) was found to be a superior suture material in a study [30]. In addition, four-strand core sutures lead to less gapping but caused more inflammatory response within the tendon [31].

Recent studies focus on using various agents to modify the healing environment. The most promising ones are TGF-*β*, NF-k*β*, and VEGF [16, 32–34]. Platelet-rich plasma had also been studied with very variable outcomes [35, 36].

Moreover, there exists lots of studies to assess the tendon adhesions either with full thickness tenotomies or direct traumas or crush injuries [7, 37–40]. The majority of these studies assess the quality and character of the tendon adhesions using macroscopic and histological grading scales; on the other hand, biomechanical data was rarely evaluated. A recent study revealed Achilles tendon model in rats as a unique technique in the assessment of adhesion formation [37]. We preferred to use a rodent to evaluate the effects of TAM on adhesion formation.

TAM is a first-generation selective estrogen receptor modulator (SERM) that acts as a competitive inhibitor for estrogen receptors [41]. It has antiestrogenic effects on breast and, at the same time, proestrogenic activity on bone in postmenopausal women preventing osteoporosis [41–43]. Some reported beneficial effects of TAM include free radical scavenger, inhibition of fibrosis, calcium modulation, stabilization of biological membranes, and prevention of apoptosis [44–46].

Tendon and ligaments play key roles on the loading of the joints. The balance between the production and the degradation of the tendon fibroblasts determines the overall metabolism; thus, homeostasis is established [47]. It is still controversial if estrogen has activity on tendons and ligaments. However, some studies exhibit the existence of estrogen receptors on those [48–51]. In one of these studies, another SERM, raloxifene, restored the downregulation of tendon collagen turnover [51].

Up to 21st century, it was not known that TAM had additional features such as antifibroblastic effects leading to reports improving scar formation [14]. It had been shown that postmenapausal women had better scar formation when compared to premenapausal women [52]. In a study, the existence of different estrogen levels of those women played critical role on high-quality scar formation [53]. Takeyama et al. [47] showed that TAM decreased the levels of TGF-*β*1 in keloid cells; on the other hand, Ruffy et al. [14] could not be able to declare an increase in TGF-*β*1 in the presence of TAM. According to the in vitro findings, TAM was found to improve scar formation [14]. A review by Meng et al. depicted TGF-*β* as the master regulator of fibrosis [54]. In this study, most of the fibrosis pathways in chronic kidney disease had been elucidated, and TGF-*β*1 had been found as the potential target to inhibit fibrosis. Karaca et al. introduced the beneficial effects of TAM on postoperative intra-abdominal adhesions [11]. They had similar findings by using low (1 mg/kg) and high (10 mg/kg) dose of TAM [11]. Moreover, TAM had become a remarkable glimmer of hope in silicosis which is widely known as a progressive scarring disease in lungs [55]. These effects possibly take place via complex actions of specific genes [56]. In another study, the effects of 200, 400, and 800 mg/kg/day TAM were investigated in rats [57]. Here, we tried to clarify the effects of TAM when administered locally and/or systematically. Therefore, a low and high dose of TAM as 1 mg/kg and 40 mg/kg per day was administered systematically, respectively. In addition, local effect of TAM was investigated with the local injection at a dose of 1 mg/kg per day.

Topical effects of TAM on rat wound healing had also been studied [58]. According to this study, local application of TAM increased angiogenesis and decreased fibrotic tissue thickness. The authors proposed that these effects expedited the wound healing process, reduced contracture, and prevented hypertrophic scar. We found similar results with these outcomes. However, we think that the least scar formation and peritendinous adhesion were ensured via local application of TAM rather than systemic administration. Thus, the biomechanical scores were more significant in groups 2 and 4 when compared to groups 1 and 3. In addition, histopathological results revealed that high-dose TAM had not yielded a significant value when compared with the low-dose counterpart.

TGF-*β* is a cytokine that has potent activities on wound healing including fibroblast and macrophage recruitment, stimulation of collagen production, downregulation of proteinase activity, and enhancement in metalloproteinase inhibitor [15, 59, 60]. All TGF-*β* isoforms increase collagen production [15]. Therefore, inhibition of TGF-*β* may control the fibrosis. TGF-*β* binds to 3 membrane peptides named RI, RII, and RII, where RI and RII are transmembrane serine/threonine receptors; on the contrary, RIII is a membrane-bound proteoglycan. TGF-*β* and these receptors are the key modulators of wound healing [15].

There are some agents that inhibit or reduce the effects of TGF-*β*, TGF-*β*1, TGF-*β*2, or TGF-*β*3 such as quercetin, tetrandrine, decorin, hepatocyte growth factor, ghrelin, CD109, tumor necrosis factor, and tamoxifen [61]. According to the recent studies, TAM decreases the expression of TGF-*β*1, TGF-*β*2, and TGF-*β*3 via non-Smad signaling through ERK1/2 [61–64]. It is proven that TAM does not interfere with Smad signaling and blocks the expression of myofibroblast marker proteins in primary human fibroblasts [63]. Since myofibroblasts excrete some cytokines and proteases, they play key role in tumor microenvironment [65]. Therefore, the investigation on the prevention of activation of myofibroblasts has provided TGF-*β* as a crucial therapeutic tool, particularly in breast cancer [63, 66].

Most of the studies show remarkable affirmative effects of TAM on wound healing, reduction of hypertrophic scar after surgery, prevention of myofibroblast differentiation, and inhibition of the effects of TGF-*β* in human fibroblasts; however, no studies were found to elucidate the effects of TAM in the prevention of tendinous adhesions [61, 63].

In our study, we constructed 4 randomized groups as control (group 1) and study groups (groups 2, 3, and 4). Group 1 was divided into 2 as control and sham. Sham group consisted of tendons in which no intervention was carried out, whereas control group included the tendons with the involvement of transection and suturation. The aim of the inclusion of sham group was to evaluate the differences among the tendons having no intervention with the ones having management as well. Each parameter was compared statistically with the relevant counterpart in order to ensure a significant outcome. Macroscopic and microscopic evaluation revealed that group 4 had the similar findings with group 1 control (G1CON) meaning that the local administration of TAM established less peritendinous adhesion like in the control group with regard to groups 2 and 3. Biomechanically, maximum force that led to tendon rupture was observed in group 2. This force was found minimum in group 3. Henceforth, the tendons in groups 2 and 3 showed the maximum and minimum strength, respectively. Following group 2, group 4 had similar tensile strength. Statistical significance was found between control and sham groups, groups 1 (control) and 2, groups 1 (sham) and 3, groups 2 and 3, groups 2 and 4, and groups 3 and 4.

There are some drawbacks in our study although this is an animal experiment. Factors that impact tendon healing such as age, activity level, body mass index, the presence of comorbidities, and smoking were discarded. All these factors have significant influences on human tendon healing [67]. The differences between the human and rodent immune systems affect the healing response of tendons [68, 69]. Nevertheless, the relationship between rodent models and human tendon healing is an important issue that that will need to be addressed in future studies and prior to clinical translation. The fundamental understanding of tendon cell biology during tendon healing is still a debate; however, the future research will reveal the unique potential of all anatomic units around the tendon with the advent of cutting-edge techniques in order to enhance more regenerative healing.

TAM is a crucial drug for patients having breast cancer. Here, a different indication of TAM is investigated. More human studies will reveal the routine use of TAM and clarify the absolute indications and contradictions.

## 5. Conclusion

Low- and high-dose administration of systemic TAM had some effects on peritendinous adhesion; however, the statistical parameters have been distributed randomly. TAM with local administration had the upmost benefit in the reduction of peritendinous adhesions, pathologically. Thus, this was proven statistically. However, the tendons in which low-dose TAM was administered showed the maximum strength biomechanically with a high statistical significance.

More human trials will reveal the use of TAM in routine tendon repairs, either in upper or lower extremity.

## Figures and Tables

**Figure 1:** (a) Isolation of Achilles tendon. (b) Division of Achilles tendon. (c) Repair of Achilles tendon with nonabsorbable suture material (polypropylene).

**Figure 2:** Tendon sample placed between jaws of tensile appliance during tendon tensile test. (a) Front view. (b) Side view.

**Figure 3:** Histopathological findings. (a) A number of scattered filaments, irregular and shortened slight adhesions (G1CON). (b) A large number of filaments, shortened, filamentous with slight adhesions (G1CON). (c) Countless, dense filaments with severe adhesions (group 2). (d) Regular, fine number of scattered filaments and slight adhesions (group 3). (e) A large number of filaments, shortened, filamentous appearance with moderate adhesions (group 3). (f) A large number of dense filaments with severe adhesions (group 3). (g) A number of scattered filaments, regular, elongated appearance with slight adhesions (group 4). (h) A large number of filaments, mixed, shortened, filamentous appearance with slight adhesions (group 4). (i) Fibroblastic activity in Masson's trichrome staining showing scattered filaments (G1CON). (j) Fibroblastic activity in Masson's trichrome staining showing dense filaments (group 2). (k) Fibroblastic activity in Masson's trichrome staining showing moderate adhesions (group 3). (l) Fibroblastic activity in Masson's trichrome staining with slight adhesions (group 4). (m) Please notice the mean loss of elastic fibers in Masson's trichrome staining (group 4). Upper two rows are stained in hematoxylin and eosin.

**Figure 4:** Mean maximum rupture force values obtained during tensile test on tendons. Groups with significant difference ^∗^*p* < 0.01.

**Figure 5:** Pathological findings revealed statistically significance between the groups with the brackets. The values in *y*-axis indicate mean measurements. Moreover, the significant values are summarized in the table at the right bottom side (CON: control; G1: group 1; G2: group 2; G3: group 3; G4: group 4; macro1: macroscopic finding quantity segment; macro2: macroscopic finding quality segment; macro3: macroscopic finding grading of adhesion segment; micro1: histopathological finding quantity segment; micro2: histopathological finding quality segment; micro3: histopathological finding grading of adhesion segment). Here, you will find the relevant statistical significance among the groups with the identical color in brackets (green: macro1; red: macro2; grey: macro3; yellow: micro1; blue: micro2; purple: micro3).

**Table 1:** Macroscopic grading system for adhesions according to Tang et al. [32].

Points	Features of adhesions
	Length (quantity)
0	No adhesions
1	<5 mm
2	5 to 10 mm
3	>10 mm
	Density and tolerance for mobility (quality)
0	No adhesions
1	Loose, elastic, and mobile
2	Moderate mobility
3	Rigid, dense, and immobile
	Grading of adhesions
0	Absent
1, 2	Slight
3, 4	Moderate
5, 6	Severe

**Table 2:** The grading criteria of adhesions in histologic evaluation according to Tang et al. [32].

Points	Features of adhesions
	Quantity
0	No apparent adhesions
1	A number of scattered filaments
2	A large number of filaments
3	Countless filaments
	Quality
0	No apparent adhesions
1	Regular, elongated, fine, and filamentous
2	Irregular, mixed, shortened, and filamentous
3	Dense, filamentous
	Grading of adhesions
0	No adhesions
1, 2	Slight adhesions
3, 4	Moderate adhesions
5, 6	Severe adhesions

**Table 3:** Macroscopical, histopathological, and adhesion mean scores among the groups. Please notice that similar findings are observed between group 2 and group 3. Group 4 shows reduced scores compared with the other groups. The generated peritendinous habitual reaction to trauma is profoundly less in group 4 when compared to G1CON (macro: macroscopical; micro: microscopical-histopathological; G1CON: group 1 control; G1SHAM: group 1 sham).

	G1CON	G1SHAM	Group 2	Group 3	Group 4
macro1 (quantity)	1.54	0.00	2.18	1.63	0.91
macro2 (quality)	1.72	0.00	1.81	2.09	1.27
macro3 (adhesion)	2.00	0.00	3.27	3.63	1.27
micro1 (quantity)	1.81	0.00	2.27	2.09	1.18
micro2 (quality)	1.90	0.00	2.09	2.09	1.18
micro3 (adhesion)	2.73	0.00	3.27	3.90	1.36

**Table 4:** Macroscopic evaluation of adhesion scores among the groups. Distribution of the animals regarding their adhesion scores. You can notice that slight adhesion was established in group 4 which is similar with the control group. On the contrary, groups 2 and 3 have adhesions ranged between slight and severe (G1CON: group 1 control; G1SHAM: group 1 sham).

	No adhesion	Slight adhesion	Moderate adhesion	Severe adhesion
G1CON		9 (82%)	2 (18%)	
G1SHAM	11 (100%)			
Group 2		4 (36%)	5 (45%)	2 (19%)
Group 3		2 (18%)	7 (64%)	2 (18%)
Group 4	1 (9%)	10 (91%)		

**Table 5:** *p* values were calculated between the groups with the same parameters. Bold ones show the statistically significant values. Please note *p* below 0.05 was established between G1CON and G1SHAM in each parameter. Moreover, most of the parameters between G1CON and group 4 showed *p* below 0.05. This table summarizes the statistics of Figure 4 (G1CON: group 1 control; G1SHAM: group 1 sham).

Groups	*p* value
G1CONmacro1 - G1SHAMmacro1	**.000**
G1CONmacro2 - G1SHAMmacro2	**.000**
G1CONmacro3 - G1SHAMmacro3	**.000**
G1CONmicro1 - G1SHAMmicro1	**.000**
G1CONmicro2 - G1SHAMmicro2	**.000**
G1CONmicro3 - G1SHAMmicro3	**.000**
G1CONmacro1 - G2macro1	**.002**
G1CONmacro2 - G2macro2	.724
G1CONmacro3 - G2macro3	**.011**
G1CONmicro1 - G2micro1	.096
G1CONmicro2 - G2micro2	.506
G1CONmicro3 - G2micro3	.237
G1CONmacro1 - G3macro1	.676
G1CONmacro2 - G3macro2	**.038**
G1CONmacro3 - G3macro3	**.000**
G1CONmicro1 - G3micro1	.082
G1CONmicro2 - G3micro2	.341
G1CONmicro3 - G3micro3	**.005**
G1CONmacro1 - G4macro1	.067
G1CONmacro2 - G4macro2	.096
G1CONmacro3 - G4macro3	**.038**
G1CONmicro1 - G4micro1	**.011**
G1CONmicro2 - G4micro2	**.024**
G1CONmicro3 - G4micro3	**.001**
G2macro1 - G3macro1	.052
G2macro2 - G3macro2	.277
G2macro3 - G3macro3	.397
G2micro1 - G3micro1	.441
G2micro2 - G3micro2	1.000
G2micro3 - G3micro3	.152
G2macro1 - G4macro1	**.005**
G2macro2 - G4macro2	.052
G2macro3 - G4macro3	**.005**
G2micro1 - G4micro1	**.001**
G2micro2 - G4micro2	**.010**
G2micro3 - G4micro3	**.002**
G3macro1 - G4macro1	**.024**
G3macro2 - G4macro2	**.020**
G3macro3 - G4macro3	**.000**
G3micro1 - G4micro1	**.005**
G3micro2 - G4micro2	**.010**
G3micro3 - G4micro3	**.000**

## Data Availability

No data were used to support this study.

## Abbreviations

TGF-*β*: Transforming growth factor-beta
NF-k*β*: Nuclear factor kappa-beta
VEGF: Vascular endothelial growth factor
EGF: Epidermal growth factor
NSAID: Nonsteroidal anti-inflammatory drug
Macro: Macroscopic
Micro: Histopathological
Number 1: Quantity
Number 2: Quality
Number 3: Grading of adhesion (e.g., macro2 means quality of adhesion macroscopically; micro3 means grading of adhesion histopathologically).
